# Stress cardiomyopathy associated with the first manifestation of multiple sclerosis: a case report

**DOI:** 10.1186/s12883-020-01757-6

**Published:** 2020-06-04

**Authors:** Daniel Rapp, Mirjam Keßler, Elmar Pinkhardt, Markus Otto, Hayrettin Tumani, Makbule Senel

**Affiliations:** 1 Department of Neurology, University of Ulm, Oberer Eselsberg 45, 89081 Ulm, Germany; 2 Department of Internal Medicine II, University of Ulm, Albert-Einstein-Allee 23, 89081 Ulm, Germany; 3 Specialty Hospital of Neurology Dietenbronn, Schwendi, Germany

**Keywords:** Multiple sclerosis, Stress cardiomyopathy, Takotsubo cardiomyopathy, Case report, Serum NfL

## Abstract

**Background:**

We present a case with a close temporal association of the first diagnosis of multiple sclerosis and stress cardiomyopathy.

**Case presentation:**

A 19-year-old man experienced severe dyspnoea. The cardiac biomarkers troponin T and NT-proBNP were elevated, and transthoracic echocardiography showed basal hypokinesia. The man was diagnosed with stress cardiomyopathy after main differential diagnoses such as acute coronary syndrome, myocarditis, and pheochromocytoma were excluded. Furthermore, the patient reported vertigo and paraesthesia. Brain and spinal MRI revealed T2-hyperintense lesions with a prominent acute lesion in the pontomedullary area. Cerebrospinal fluid findings revealed a lymphocytic pleocytosis and intrathecal IgG synthesis. Serum neurofilaments were elevated. The patient was diagnosed with MS, and treatment with intravenous Methylprednisolone was initiated. The brainstem lesion due to multiple sclerosis was assumed to be the cause of stress cardiomyopathy. The patient fully recovered.

**Conclusion:**

Stress cardiomyopathy may be linked with the first manifestation of multiple sclerosis in the presented case since pontomedullary lesions could affect the sympathetic nervous system. This case highlights the importance of neurological history and examination in young patients with unexplained acute cardiac complaints.

## Background

Stress cardiomyopathy (also takotsubo cardiomyopathy or broken-heart syndrome) is a transient loss of function of the left ventricle with characteristic wall-motion abnormalities. The most common form presents as apical ballooning [1] due to akinetic left ventricular apex. The clinical presentation, electrocardiogram (ECG) abnormalities, and elevated heart-specific biomarkers mimic acute coronary syndrome. Here, we present a case of stress cardiomyopathy in a young man associated with the first diagnosis of multiple sclerosis (MS).

## Case presentation

A 19-year-old man without medical history experienced severe dyspnoea and was admitted to hospital as an emergency. The patient negated angina pectoris. Initial blood pressure was high (240/110 mmHg), an ECG showed no relevant abnormalities, but cardiac biomarkers troponin T and NT-proBNP were elevated (27-fold (372 ng/L), and 26-fold (2225 pg/mL) of the upper normal limit (UNL), respectively). Transthoracic echocardiography showed impaired left ventricular function with basal hypokinesia. Treatment with Nebivolol and Candesartan was initiated. Cardiac magnetic resonance imaging (MRI) at day 3 showed no evidence of acute myocarditis. The left ventricular function had recovered at that time. Coronary angiography showed no evidence of coronary heart disease, thus excluding myocardial infarction as the reason for troponin T elevation and basal left ventricular hypokinesia. Endocarditis was excluded by transthoracic and transoesophageal echocardiography and repeated blood cultures. Normal blood levels of catecholamines and metanephrines excluded pheochromocytoma. The cardiac biomarkers decreased over follow-up (Fig. 1).

**Fig. 1:** Heart-specific biomarkers and serum neurofilaments Timeline of biomarkers showing multiples of the upper normal limit (UNL) in the course of the hospital stay sNfL = serum neurofilaments, BNP = brain natriuretic peptide. (*) brain MRI performed (§) lumbar puncture performed (†) intravenous Methylprednisolone (1 g/day for five days). Troponin and NT-pro BNP are shown in multiples of the upper normal limit (UNL, Troponin T 14 ng/L, Troponin I 0.026 ng/mL, NT-pro BNP 85.8 pg/mL). Troponin T from admission until day 3 and Troponin I on day 6

After the acute phase, the patient complained about vertigo. The neurological examination showed upbeat nystagmus, hyperreflexia of the lower limbs, as well as unsteady gait. On specific demand, the patient reported that he had experienced paraesthesia of the entire left side of the body and as well in the right arm and leg since 5 days before admission to the hospital. Brain and spinal MRI were performed, showing supra- and infratentorial, as well as spinal T2-hyperintense lesions (Fig. 2). One prominent lesion was found in the pontomedullary area, showing Gadolinium-enhancement and a high signal in diffusion-weighted imaging (DWI) (Fig. 2 E-H). Cerebrospinal fluid (CSF) analysis revealed a lymphocytic pleocytosis (13 leucocytes per μL), and CSF specific oligoclonal IgG bands. Screening of potential other autoimmune or infectious diseases was negative. Serum neurofilament (sNfL) levels (measured using single-molecule array technology) were elevated while troponin T levels were still over the UNL (Fig. 1). Serum-Aquaporin-4- and -MOG-antibodies were negative. Evoked potential latencies showed lesions in the somatosensory pathway of the left leg as well as in the visual pathway of the right eye. The patient was diagnosed with MS according to current criteria [2] and treatment with intravenous methylprednisolone (1 g/day for 5 days) was initiated. During the hospital stay, the patient fully recovered and showed no focal signs at the time of discharge. A disease-modifying treatment with Teriflunomide (14 mg/day) was initiated. In follow-up examinations, 5 months later, the patient showed no abnormalities in the stress-ECG and echocardiography. Furthermore, the patient reported no events suspicious of a relapse in the first 6 months of follow-up.

**Fig. 2:** Brain-MRI shows multiple supratentorial (**a**-**c**) and infratentorial (**d**-**h**), as well as one spinal (not shown) lesions suggestive of multiple sclerosis. The lesion in the medulla oblongata (**e**-**g**) (12x10mm) shows Gd-enhancement and high signal on DWI. A,B,D transverse T2 TSE, C,E sagittal T2 TSE, F transverse DWI weight, G coronal T2-FLAIR, H coronal T1 VIBE

## Discussion and conclusions

We report a patient presenting with stress cardiomyopathy and subsequent diagnosis of MS. An extensive diagnostic work-up including ECG, echocardiography, cardiac MRI, coronary angiography, and serology, excluded main differential diagnoses, such as acute coronary syndrome, myocarditis, and pheochromocytoma. No other cause of stress cardiomyopathy was found except for an acute demyelinating pontomedullary lesion identified as the first manifestation of MS.

The exact pathophysiological mechanisms for stress cardiomyopathy are not fully understood. Unlike ischemic myocardial infarction, stress cardiomyopathy is assumed to be triggered by high levels of catecholamines as a result of emotional stress or an excessive endogenous secretion [1]. Recently, some case studies have reported a coincidence of brainstem lesions due to MS and stress cardiomyopathy [3–6]. Consistent with this, MRI imaging of the case described here revealed an acute pontomedullary Gd-enhancing lesion. It is known that some areas which regulate the autonomous nervous system are located in this area of the brainstem [7]. Pontomedullary lesions may thereby cause excessive catecholamine secretion and lead to an increased vulnerability for stress cardiomyopathy. A direct increase of Troponin by a brainstem lesion seems unlikely [8]. Furthermore, not only troponin as a heart-specific marker but also sNfL, a widely accepted marker for neuroaxonal injury [9, 10] detected by the single-molecule array technology, were elevated.

In conclusion, prospective studies are needed to confirm the hypothesis of increased risk for stress cardiomyopathy in MS patients. However, as a consequence of the mentioned cases, we recommend obtaining a detailed neurological history and examination in young patients with unexplained acute cardiac complaints.

## Data Availability

The datasets used and/or analysed during the current study are available from the corresponding author on reasonable request.

## Abbreviations

CSF: Cerebrospinal fluid
DWI: Diffusion-weighted imaging
ECG: Electrocardiography
Gd: Gadolinium
MRI: Magnetic resonance imaging
MS: Multiple sclerosis
NT-proBNP: N-terminal pro-B-type natriuretic peptide
sNfL: Serum Neurofilament
UNL: Upper normal limit
